The article "Phytochemical Analysis and Antioxidant, Antibacterial, and Antifungal Effects of Essential Oil of Black Caraway (Nigella sativa L.) Seeds against Drug-Resistant Clinically Pathogenic Microorganisms" was published in 2022. Journal: Biomed Res Int.

# Phytochemical Analysis and Antioxidant, Antibacterial, and Antifungal Effects of Essential Oil of Black Caraway (*Nigella sativa* L.) Seeds against Drug-Resistant Clinically Pathogenic Microorganisms

**DOI:** 10.1155/2022/5218950

**Published:** 2022-07-26

**Authors:** Otmane Zouirech, Abdullah A. Alyousef, Azeddin El Barnossi, Abdelfattah El Moussaoui, Mohammed Bourhia, Ahmad M. Salamatullah, Lahcen Ouahmane, John P. Giesy, Mourad A. M. Aboul-soud, Badiaa Lyoussi, Elhoussine Derwich

**Affiliations:** ^1^Laboratory of Natural Substances, Pharmacology, Environment, Modeling, Health and Quality of Life (SNAMOPEQ), Faculty of Sciences Dhar El Mahraz, University Sidi Mohamed Ben Abdellah, Fez, Morocco; ^2^Department of Clinical Laboratory Sciences, College of Applied Medical Sciences, King Saud University, P.O. Box 10219, Riyadh 11433, Saudi Arabia; ^3^Laboratory of Biotechnology, Environment, Agrifood, and Health, Faculty of Sciences Dhar El Mahraz, University of Sidi Mohamed Ben Abdellah, Fez 30050, Morocco; ^4^Laboratory of Microbial Biotechnology, Agro-Sciences and Environment (BioMAgE), Cadi Ayyad University, Marrakesh 40000, Morocco; ^5^Department of Food Science & Nutrition, College of Food and Agricultural Sciences, King Saud University, P.O. Box 2460, Riyadh 11451, Saudi Arabia; ^6^Department of Veterinary Biomedical Sciences & Toxicology Centre, University of Saskatchewan, Saskatoon, SK, Canada S7N5B3; ^7^Department of Environmental Science, Baylor University, Waco, TX 76798-7266, USA; ^8^Unity of GC/MS and GC-FID, City of Innovation, Sidi Mohamed Ben Abdallah University, Fez, Morocco

## Abstract

*Nigella sativa* (NS) is a plant that has long been utilized in traditional medicine as a treatment for certain diseases. The aim of this work was to valorize the essential oil (EO) of this species by phytochemical analysis and antimicrobial and antioxidant evaluation. EO was extracted by hydrodistillation from the seeds of *Nigella sativa* (EO-NS). Phytochemical content of EO-NS was evaluated by use of gas chromatography coupled to mass spectrometry (GC-MS/MS). Antioxidant ability was *in vitro* determined by use of three assays: 2.2-diphenyl-1-picrylhydrazyl (DPPH), ferric reducing power (FRAP), and total antioxidant capacity (TAC) relative to two synthetic antioxidants: BHT and quercetin. Antimicrobial effect was evaluated against four clinically important bacterial strains (*Staphylococcus aureus*, ATCC 6633; *Escherichia coli*, K12; *Bacillus subtilis*, DSM 6333; and *Proteus mirabilis*, ATCC 29906) and against four fungal strains (*Candida albicans*, ATCC 10231; *Aspergillus niger*, MTCC 282; *Aspergillus flavus*, MTCC 9606; and *Fusarium oxysporum*, MTCC 9913). Fifteen constituents that accounted for the majority of the mass of the EO-NS were identified and quantified by use of GC-MSMS. The main component was *O*-cymene (37.82%), followed by carvacrol (17.68%), *α*-pinene (10.09%), trans-sabinene hydrate (9.90%), and 4-terpineol (7.15%). EO-NS exhibited significant antioxidant activity with IC_50_, EC_50_, and total antioxidant capacity (TAC) of 0.017 ± 0.0002, 0.1196 ± 0.012, and 114.059 ± 0.97 mg EAA/g, respectively. Additionally, EO-NS exhibited promising antibacterial activity on all strains under investigation, especially on *E. coli* K12 resulting in inhibition diameter of 38.67 ± 0.58 mm and a minimum inhibitory concentration (MIC) of 1.34 ± 0.00 *μ*g/mL. Also, EO-NS had significant antifungal efficacy, with a percentage of inhibition of 67.45 ± 2.31% and MIC of 2.69 ± 0.00 *μ*g/mL against *F. oxysporum*, MTCC 9913 and with a diameter of inhibition 42 ± 0.00 mm and MIC of 0.67 ± 0.00 *μ*g/mL against *C. albicans*. To minimize development of antibiotic-resistant bacteria, EO-NS can be utilized as a natural, alternative to synthetic antibiotics and antioxidants to treat free radicals implicated in microbial infection-related inflammatory reactions.

## 1. Introduction

Excessive generation of free radicals damages biological components directly by oxidation of DNA, proteins, lipids, and carbohydrates, as well as causing secondary damage, due to cytotoxic and mutagenic effects of metabolites released [1]. Due to the diversity and severity of medical problems caused by oxidative stress [2], and the fact that use of synthetic antioxidants is no longer recommended because of their carcinogenic potential [3], in order to minimize oxidative stress and its associated pathologies, new antioxidants have been sought [4]. In particular, natural products of plants are regarded as having potential as antioxidant compounds for protection of cells against damage caused by free radicals [5, 6].

Antimicrobial resistance (AMR) is a major and ongoing global challenge and a threat to public health. It is estimated that by 2050, AMR will be responsible for ten million deaths with a total cost of 100 trillion dollars [7]. Faced with this problem, alternative therapeutic solutions, based on natural resources, particularly medicinal plants, have been the subject of extensive research to develop new antibiotics or new therapeutic modalities and to seek alternatives to currently used antibiotics and develop alternative molecules effective against infectious diseases [8–10]. Aromatic and medicinal plants are an important source of bioactive compounds, such as essential oils (EOs) that could be applied as therapies for infectious diseases [11–14]. EOs have been shown to be valuable as a nontraditional sources of natural, bioactive antioxidants and antimicrobials to combat antibiotic-resistant bacteria and harmful reactive oxygen species (ROS) and are involved in inflammatory immune responses associated with infection. EO derived from seeds of black caraway *Nigella sativa*, a flowering plant in the family Ranunculaceae (EO-NS), was recently studied for biological activities [15, 16]. *N. sativa* is also often referred to as black cumin, nigella, or kalonji. The aim of the current study was to examine the chemical composition of EO-NS as well as their antioxidant and antimicrobial potential against antibiotic-resistant pathogenic and phytopathogenic microorganisms.

## 2. Materials and Methods

### 2.1. Plant Material

Seeds of the black caraway (*N. sativa*) were collected in the Souk El Arbaa area of Morocco (34°39′57 ″N 5°58′54 ″W).

### 2.2. Extraction and Identification of Constituents of EO-NS

The EO of the crushed seeds was extracted through hydrodistillation for a period of 4 h at 100°C by use of Clevenger apparatus (Haborne, 1984) [17]. The chemical profiling of EO-NS was conducted by GC coupled to spectrometer. Varian capillary was employed (Model: TR5- CPSIL-5CB) with length, diameter, and film thickness of 50 m, 0.32 mm, and 1.25 *μ*m, respectively. Temperature programming of the column was in the range of 45-290°C increasing with a steady rate of 4°C/min. While the injector had a fixed temperature of 280°C, temperature of the detector (MS-PolarisQ) was 200°C. The flow rate of helium (carrier gas) was set to 1 mL/min. The injection volume for EO was 1 *μ*L, after having been diluted in organic solvent (hexane) according to the technique of splitless injection. In electronic ionization mode, the ionization energy was 70 eV. The ion source and interface temperatures were 200°C and 350°C, respectively. The range employed for scanning mass was 30-650 m/z. Identification of EO-NS phytoconstituents was conducted by the comparison of their Kovats index values, which were calculated compared to the retention times of a group of linear alkanes (C4-C29), with the values of those standard references collected by Adams library and NIST-MS V2.0 search.

### 2.3. *In Vitro* Antioxidant Activity of EO-NS

#### 2.3.1. DPPH Assay

Antioxidant effects of EO-NS were evaluated by use of previously published methods [18]. Briefly, 800 *μ*L of DPPH (0.2 mM, in methanol) was added to 200 *μ*L of various serial dilutions of EO-NS ranging from 0 (in the control) to 1 mg/mL. The obtained mixture was then kept in the dark for 30 min at room temperature (RT). Absorbances were measured at 517 nm against a control consisting of 800 *μ*L of DPPH and methanol solution. Positive controls of quercetin or BHT and blank control were prepared under the same conditions. Antioxidant activity was expressed as percent of inhibition (PI) of the absorbance at 517 nm.

(1) $$\begin{array}{c} \text{PI}\left(\%\right)=\left(1-\frac{\text{Sample absorbance}}{\text{Control absorbance}}\right)*100. \end{array}$$

The IC_50_ is the concentration of either EO-NS or ascorbic acid, necessary to reduce free radicals in the reaction medium by 50%. The abscissa represents the concentration values of the tested compound and the ordinate represents the percentage inhibition, with IC_50_ values obtained by linear regression and interpolation (PI%).

#### 2.3.2. Total Antioxidant Capacity (TAC)

The total antioxidant capacity (TAC) of EO-NS was measured by use of the phosphomolybdenum method. Briefly, 100 *μ*L of various concentrations of EO-NS was added to 1000 *μ*L of H_2_SO_4_, Na_2_PO_4_, and ammonium molybdate reagent mixture such that their concentration was in the range of 0.6 M, 28 mM, and 4 mM, respectively. The tubes were placed at a temperature of about 95°C for 90 minutes. After cooling, the absorbance was read at 695 nm. The control consisted of 100 *μ*L of methanol mixed with 1000 *μ*L of reagent mixture [19]. Samples and controls are incubated under identical conditions. The results obtained are represented as mg of ascorbic acid equivalents per gram (mg EAA/g).

#### 2.3.3. Reduced Ferric Assay (FRAP)

The ferric reduction process relies on antioxidants to reduce ferric iron to iron salt, which results in formation of a blue solution. Briefly, 200 *μ*L of different concentrations of EO-NS and 500 *μ*L of 0.2 M phosphate buffer (pH 6.6) were added to glass tubes, followed by 500 *μ*L of 1% potassium hexacyanoferrate (K_3_Fe(CN)_6_) in distilled water. The mixture was heated to 50°C for 20 minutes in a water bath. A 500 *μ*L volume of trichloroacetic acid (10%) was pipetted, and the solution was subjected to centrifugation at 3000 rpm for 10 min. A 500 *μ*L aliquot of the supernatant was transferred to another tube to which 500 *μ*L of double-distilled water (ddH_2_O) and 100 *μ*L of 1% FeCl_3_, freshly prepared, in ddH_2_O were added. A blank without an EO sample was also prepared similarly by replacing the EO-NS with methanol. The absorbance was read at 594 nm with reference to the blank, replacing the EO-NS with methanol, which allows calibrating the apparatus (UV-VIS spectrophotometer). Solution of standard antioxidants, either BHT or quercetin, whose absorbances were read in a similar fashion as with the samples, served as positive controls [20].

### 2.4. *In Vitro* Antimicrobial Activity of EO-NS

#### 2.4.1. Microbial Strains

The antimicrobial capacity of EO-NS was assessed against four clinically important fungal strains (*Candida albicans*, ATCC 10231; *Aspergillus niger*, MTCC 282; *Aspergillus flavus*, MTCC 9606; and *Fusarium oxysporum*, MTCC 9913) and four bacterial strain (*Staphylococcus aureus*, ATCC 6633; *Escherichia coli*, K12; *Bacillus subtilis*, DSM 6333; and *Proteus mirabilis*, ATCC 29906), which were obtained by Sidi Mohammed Ben Abdellah University (Fez, Morocco).

#### 2.4.2. Method for Assessing Antimicrobial Activity

Antimicrobial activity of EO-NS was assessed by use of the disc diffusion method [21]. Briefly, Petri dishes containing Mueller-Hinton and malt extract were inoculated with the four bacterial strains and *C. albicans*, respectively, using the double-layer method. From fresh cultures grown in Mueller-Hinton and malt extract media, serial dilutions were established in sterilized saline solution (NaCl, 0.9%) until obtaining turbidity of 0.5 McFarland (10^6^ to10^8^ CFU/mL). Then, 100 *μ*L was added to tubes containing 5 mL of soft agar (0.5% agar), and the inoculated tubes were plated into Petri dishes containing Mueller-Hinton and malt extract media. Whatman paper discs No. 4, with a diameter of 6 mm, were impregnated with 20 *μ*L of EO-NS. For the fungal strains *A. niger*, *A. flavus*, and *F. oxysporum*, the antifungal potency was determined by use of the direct confrontation assay in the malt extract medium between EO-NS and the fungal strains tested. Briefly, Whatman paper discs No. 4 with a diameter of 6 mm were soaked with 20 *μ*L of EO-NS, and an agar plate of the fungal strain was positioned 1 cm from the disc containing EO-NS. To assess the efficacy of EO-NS negative controls and positive controls containing conventional antimicrobial drugs, streptomycin and oxacillin for bacterial strains and fluconazole for fungal strains were performed in the same way as the tests. Petri dishes, which had been inoculated with the strain, were placed in an incubator at 30°C or 37°C for fungi or bacteria and *C. albicans*, respectively. Diameters and percentages of inhibition were measured after 24 h, bacteria; 48 h, *C. albicans*; and 7 days, *A. niger*, *A. flavus*, and *F. oxysporum* [22, 23].

#### 2.4.3. Minimum Inhibitory Concentration

Minimum inhibitory concentration (MIC) of EO-NS against each of the four strains of bacteria and fungi was determined by use of previously described methods for microdilution [23]. Briefly, sterile 96-well microplates were premarked, under aseptic conditions; then, 100 *μ*L of EO-NS prepared in DMSO (10%, *v*/*v*) was added to the first row of the plate. The following volumes were subsequently pipetted into all remaining wells, 50 *μ*L sterile Mueller-Hinton and 50 *μ*L sterile malt extract for bacterial and fungal strains, respectively. Multichannel pipette was utilized to make serial dilutions. Finally, 30 *μ*L of bacterial or fungal suspensions of each strain was pipetted into each well. Following a 24 h of incubation for bacteria, 48 h for *C. albicans*, and 7 days for *A. niger*, *A. flavus*, and *F. oxysporum* at 37°C and 30°C, respectively [21–23], the MIC end point was assessed by close observation of the growth inside the wells or *via* colorimetric determination (0.2% TTC, *w*/*v*) [23].

### 2.5. Statistical Analysis

Results were represented as means of triplicates ± standard deviation (SD). GraphPad Prism (version.8.0.1) was utilized to perform statistical analyses by use of the Shapiro-Wilk tests to verify the normality of the variables as well as Levene's test to assess the homogeneity of variances. Statistical differences between the means were calculated by analysis of variance (One way-ANOVA) and Tukey's test for multiple comparison. Significance of differences was considered at a probability cut-off level of *p* ≤ 0.05.

## 3. Results and Discussion

### 3.1. Extraction of EO-NS

The yield of EO achieved by the hydrodistillation, expressed on mass of seed, was about 0.8 ± 0.02%, with characteristic transparent yellow color with aromatic odor. This yield was similar to that of 0.832 ± 0.025% found previously for EO-NS from Beni Mellal, Morocco [24]. Several studies have the EO-NS content of *N. sativa* seeds [25] and revealed that EO-NS extracted by hydrodistillation was about 0.08%, while EO-NS extracted by microwave distillation was approximately 0.11%. Yields of EO-NS of seeds of *N. sativa* from five different countries, namely, Saudi Arabia, Syria, Morocco, India, and France, were achieved by hydrodistillation ranging from 0.047% to 1.7% [26, 27]. Variability among yields of EO-NS can be ascribed for slight differences in extraction procedures as well as other factors, such as geographic origin, ecological factors, agronomic practices, and storage conditions [27–29].

### 3.2. GC-MS/MS Studies

Based on GC-MS/MS analysis of EO-NS extracted from seeds of Moroccan origin, the following compounds and respective proportions of the total mass of EO-NS were determined. Among the 15 compounds identified, 10 were basic monoterpenoids, which accounted for 85.51% of total masses of constituents. These are mainly terpenoid hydrocarbons, including *α*-pinene, *β*-pinene, sabinene, *γ*-terpinene, *α*-terpinene, and *O-*cymene. Terpenoid alcohols represented 6.52% of total constituents EO-NS, with terpinene-4-ol and linalool comprising 5.98% and 0.54%, respectively. Terpenoid phenols, including carvacrol comprised 14.82%. Other components of EO-NS were chrysanthenyl acetate, trans and cis-sabinene hydrate, two sesquiterpenoids, which represented 2.50% of total mass of EO-NS, including longifolene and widdrol that accounted for 0.55% and 1.95%, respectively. Monoterpenes were dominant, with *O*-cymene being the major component in EO-NS of Moroccan origin. The chemical components of EO-NS and structures of main constituents of EO-NS are presented (Table 1 and Figure 1) and GC-MS/MS chromatograms (Figure 2).

### 3.3. Antioxidant Activity of EO-NS

#### 3.3.1. DPPH Assay

EO-NS exhibited significant antioxidant activity against the DPPH free radical, which was used to evaluate its antiradical efficacy (Figures 3 and 4), exhibiting an IC_50_ value of 0.017 ± 0.001 mg/mL, compared to BHT or quercetin which exhibited IC_50_ values of 0.0118 ± 0.007 and 0.035 ± 0.004 mg/mL, respectively. In comparison, the IC_50_ values of the EO-NS studied showed a greater antioxidant capacity than [30, 31] exhibiting IC_50_ values of 36.90 *μ*g/mL and 19 ± 0.7 *μ*g/mL, respectively.

Various components in EOs, including terpenes, sesquiterpenes, and phenolic compounds, which function in diverse modes, can be linked to their antioxidant properties. The principal phytoconstituents EO-NS were *O*-cymene, carvacrol, 4-terpineol, and longifolene, which were responsible for antioxidant properties of EO-NS [15, 32, 33].

#### 3.3.2. FRAP Assay

Results of the FRAP assay revealed that EO-NS exhibited significant dose-dependent, reducing activity exhibiting an EC_50_ of 0.119 ± 0.013 mg/mL (Figure 4). This potency was comparable with that of BHT with EC_50_ of 0.139 ± 0.0110 mg/mL, but less than that of quercetin with an EC_50_ of 0.040 ± 0.002 mg/mL. Reducing power of EO-NS was probably due to the presence of chemically bioactive compounds. Indeed, results of previous studies on reducing power of EO-NS revealed that EO-NS possess considerable reducing power [30, 34]. Specifically, the reducing power of EO-NA can be attributed to phenolic compounds especially carvacrol, which have a hydroxyl-OH group that can donate a hydrogen atom [35, 36]. Other chemicals that operate synergistically with EOs, such as alcohols (linalool), ethers, and hydrocarbons (*α*-terpinene and *γ*-terpinene), can contribute to their antioxidant potency. [37–39].

#### 3.3.3. Total Antioxidant Capacity (TAC)

Based on results of the TAC assay, EO-NS exhibited antioxidant activity equivalent to 114.059 ± 0.972 *μ*g EAA/mg EO-NS (Figure 5). This result can be attributed to the presence of active antioxidant substances [40]. The antioxidant activity is probably attributed to the monoterpene compounds in essential oils [41]. Generally, EOs with greater terpene content possess powerful antioxidant potential [42]. Indeed, EO-NS seem to be effective antioxidant [31]. However, minor compounds are more likely than the major compounds to provide a pivotal role in the observed antioxidant potency [43]. It is well documented that synergies between various chemicals must be taken into consideration when predicting their biological activities [44, 45].

### 3.4. Antibacterial Activity of EO-NS

The *N. sativa* EO-NS exhibited measurable antibacterial efficacy against all bacterial strains tested (Figures 6 and 7) (Table 2) and showed promising antibacterial activity compared to two commercially available antibiotics (streptomycin and oxacillin), especially against *E. coli* K12 with a diameter of inhibition of 38.67 ± 0.58 mm and a MIC of 1.34 ± 0.00 *μ*g/mL. Differences in inhibition diameters obtained could be due to differences in chemical compositions of the EO, and the antibacterial activity could be due mainly to the majority compound (*O-cymene*) or to a combination of less predominant compounds found in EO-NS. Results of several studies have indicated that EOs from *N. sativa* and their single compounds are effective against infections caused by bateria. Results of the current study reported here are in agreement with those of Harzallah et al. [46], which demonstrated that EO-NS from *N. sativa* collected in Tunisia and its bioactive compound, thymoquinone, had significant antibacterial activity. Other studies have found that the seed extract derived from *N. sativa* has strong antibacterial potency against *B. subtilis*, IMG 22 with an inhibition diameter of 27 mm, against *E. coli* DM with an inhibition diameter of 19.3 mm [47]. Another study found that *N. sativa* extract has antibacterial activity against *S. aureus* (ATCC 103207) with an inhibition diameter of 19 mm and against *B. subtilis* (ATCC 27853) with an inhibition diameter of 26 mm and against *E. coli* (ATCC 12079), with an inhibition diameter of 21 mm [48]. The results presented here demonstrate greater than that or the previous studies [49], which found that ethyl alcohol extract of *N. sativa* exhibited antibacterial potency against *B. subtilis* with an inhibition diameter of 7 mm. The results of the study presented here are also more potent than that reported previously [32], which indicated that the antibacterial potency of EO-NS was greater on *S. aureus* (MTCC 9542) with an inhibition diameter of 16 mm than *Vibrio harveyi* (MTCC 7771) with an inhibition diameter of 5 mm for the 10 mg/mL concentration. EO-NS exhibits potent antibacterial activities against antibiotic-resistant bacterial strains (gram-negative and gram-positive), thereby advocating the utility of the bioactive molecules contained in EO-NS as an alternative to commercially available antibiotics to combat bacterial resistance.

The antibacterial potency of EO-NS on the bacterial strains that we have highlighted in this study is supported by literature data showing the action of EOs rich in carvacrol, whose antimicrobial efficacy is explained by the actual position of the hydroxyl group on the phenolic structure of these molecules [50–52] and which modify permeability and cause leaking of intracellular components through the specific binding to the amine and hydroxylamine groups of bacterial membrane-bound proteins [53]. Because of their cheap cost, biocompatibility, antibacterial and resistance reversal potential, lack or low toxicity to eukaryotic cells, and decreased toxicity to eukaryotic cells and the environment, these volatile compounds are termed green antimicrobials [54]; as a result, they are regarded as an efficient approach for addressing AMR in underdeveloped nations as well as in bacterial strains, including ESKAPEE members [54].

#### 3.4.1. Antifungal Activity of EO-NS

Evaluation of the *in vitro* antifungal activity of EO-NS against *A. niger*, *A. flavus*, *F. oxysporum*, and *C. albicans* by the disc diffusion method has revealed promising antifungal activity with an inhibition percentage of 67.45 ± 2.315% and MIC of 2.69 ± 0.00 *μ*g/mL against *F. oxysporum*, MTCC 9913 and with an inhibition diameter of 42 ± 0.00 mm and MIC of 0.67 ± 0.00 *μ*g/mL against *C. albicans*, compared to the control and the antibiotic fluconazole (Table 3 and Figure 8). Furthermore, EO-NS exhibits fungicidal efficacy against both *F. oxysporum* and *C. albicans*. However, EO-NS did not exhibit significant antifungal potency against *A. niger*, MTCC 282 or *A. flavus*, MTCC 9606. The current results indicated that EO-NS has an inhibitory effect against pathogenic and phytopathogenic fungi, which might be attributed for its chemical composition, especially the presence of *O-cymene*, *carvacrol, α-thujene*, and *trans-sabinene hydrate*, all of which exhibit significant antifungal efficacies [55, 56]. The significant antifungal activity against *C. albicans* might be due to the presence of *O-cymene*, a conclusion that is in agreement with results of previous studies [57, 58], which reported that *O-cymene* component of EO-NS presents antifungal potency on *C. albicans* and other pathogenic fungal strains. The results reported here are different from those of Khosravi et al. [59], which showed that EO-NS exhibits antifungal activity against *A. flavus*. For cytotoxicity of EO-NS, the study of Mahmoud et al. [60] demonstrates that EO-NS did not show significant cytotoxicity on macrophages, and results of the current study indicate promising antifungal activity of EO-NS without causing cytotoxicity, which suggests its usage as a good alternative to substitute commercially available antifungals to combat fungal resistances.

## 4. Conclusion

The results of the present study show that EO-NS was effective as antioxidants, antibacterial, and antifungal that could be used as an alternative to currently available synthetic molecules. Notably, GC/MS-MS analysis of EO-NS revealed the richness of these oils in potentially bioactive compounds with a dominance of O-cymene and carvacrol. The antioxidant activity of EO-NS was confirmed by three tests (DPPH, FRAP, and TAC) even at low concentrations. EO-NS acts as a promising antibacterial agent on almost all the studied strains, with a more pronouncing effect on *E. coli (K12)*. Antifungal activity indicated that EO-NS had broad spectrum of action against almost all the studied strains. In further studies, the focus will be on testing purified compounds of EO-NS along with investigating their mode of action. Prior to any prospective application of EO-NS as a natural agent to control microorganisms, we expect to assess the possible adverse consequences on nontarget creatures, as well as clinical trials on both humans and nonhuman primates.

## Figures and Tables

**Figure 1:** Structures of four of the major phytoconstituents of essential oil extracted from seeds of black caraway *Nigella sativa* (EO-NS).

**Figure 2:** GC-MS/MS chromatogram of essential oil extracted from seeds of black caraway *Nigella sativa* (EO-NS).

**Figure 3:** Antiradical activity of essential oil derived from seeds of *Nigella sativa* (EO-NS), by DPPH test (a), and IC_50_ values of antiradical activity of EO-NS and BHT and quercetin (b).

**Figure 4:** EC_50_ of ferric-reducing antioxidant power (FRAP) values of essential oil derived from seeds of black caraway *Nigella sativa* (EO-NS) and controls (BHT or quercetin).

**Figure 5:** Total antioxidant capacity (TAC) of essential oils extracted from seeds of black caraway *Nigella sativa* (EO-NS) and controls (BHT or quercetin).

**Figure 6:** *In vitro* antibacterial activity of essential oil extracted from seeds of black caraway *Nigella sativa* (EO-NS).

**Figure 7:** Antibacterial potency of essential oil extracted from seeds of black caraway *Nigella sativa* (EO-NS). Means (± SD, *n* = 3) with the same letter denote no evident significant differences based on Tukey's multiple range tests *p* ≤ 0.05.

**Figure 8:** *In vitro* antifungal activity of essential oil extracted from seeds of black caraway *Nigella sativa* (EO-NS).

**Table 1:** Phytochemical constituents of essential oil extracted from seeds of black caraway *Nigella sativa* (EO-NS).

P	R.T	Name	C.C	RI		Area (%)
				*Cal*	*Lit*	
1	7.68	*α*-Thujene	MO	902	930	10.09
2	7.90	*α*-Pinene	MO	948	939	2.57
3	9.03	*α*-Phellandrene	MO	994	1002	0.97
4	9.19	*β*-Pinene	MO	972	979	2.33
5	10.35	*α*-Terpinene	MO	998	1017	0.95
6	10.59	O-cymene	MO	1042	1026	46.36
7	10.72	Cis-chrysanthenyl acetate	O	1256	1265	2.56
8	11.60	Limonene	MO	998	1029	0.90
9	12.74	Cis-sabinene hydrate	O	1040	1070	0.72
10	12.81	Linalool	MO	1082	1096	0.54
11	13.43	Trans-sabinene hydrate	O	1070	1098	8.71
12	15.26	Terpinen-4-ol	MO	1148	1177	5.98
13	18.56	Carvacrol	MO	1274	1299	14.82
14	21.66	Longifolene	ST	1398	1390	1.95
15	38.23	Widdrol	ST	1604	1599	0.55
Chemical classes (C.C)						
Monoterpene (MO)						85.51
Sesquiterpene (ST)						2.50
Others (O)						11.99
Total						100

P: peak; R.T: retention time; C.C: chemical classes; RI: retention index; Cal: calculate; Lit: literature; O: others; MO: monoterpene; ST: sesquiterpene.

**Table 2:** Minimum inhibition concentration (MIC) of essential oil extracted from seeds of black caraway *Nigella sativa* (EO-NS).

	*Staphylococcus aureus* ATCC 6633	*Escherichia coli* K12	*Bacillus subtilis* DSM 6333	*Proteus mirabilis* ATCC 29906
EO-NS (*μ*g/mL)	2.69 ± 0.00^a^	1.34 ± 0.00^b^	1.34 ± 0.00^b^	2.69 ± 0.00^a^
Streptomycin (*μ*g/mL)	1.56 ± 0.00	Rs	Rs	Rs

Means (± SD, *n* = 3) labeled with different letters in same row are considered significantly different according to one-way ANOVA and Tukey's test; *p* ≤ 0.05).

**Table 3:** Antifungal activity and the MIC of essential oils extracted from seeds of black caraway *Nigella sativa* (EO-NS).

		*Candida albicans ATCC 10231*	*Aspergillus niger MTCC 282*	*Aspergillus flavus MTCC 9606*	*Fusarium oxysporum MTCC 9913*
EO-NS					
Antifungal activity		42 ± 0.00 mm^a^	0.0 ± 0.0%^b^	0.0 ± 0.0%^b^	67.45 ± 2.315%^c^
CMI (*μ*g/mL)		0.67 ± 0.00^a^	—	—	2.69 ± 0.00^b^
Fluconazole					
Antifungal activity		0.0 ± 0.0 mm^a^	8.20 ± 2.02%^b^	0.0 ± 0.0%^a^	30.77 ± 0.58%^c^
CMI (*μ*g/mL)		—	7.125^a^	—	3.125^b^

Means (± SD, *n* = 3) labelled by different letters within the same row are considered significantly different (one-way ANOVA; Tukey's test, *p* ≤ 0.05).

## Data Availability

Data used to support the findings are included within the article.
